# Low birth weight: causes and consequences

This article has been retracted.

**DOI:** 10.1186/1758-5996-5-49

**Published:** 2013-09-02

**Authors:** Carlos Antonio Negrato, Marilia Brito Gomes

**Affiliations:** 1 Department of Internal Medicine, Bauru’s Diabetics Association, 17012-433 Bauru São Paulo,Brazil; 2 Department of Internal Medicine, Diabetes Unit, State University Hospital of Rio de Janeiro, Rio de Janeiro, Brazil

## Abstract

During our phylogenetic evolution we have selected genes, the so called thrifty genes, that can help to maximize the amount of energy stored from every consumed calorie. An imbalance in the amount of stored calories can lead to many diseases. In the early 80’s the distinguished English epidemiologist David Barker, formulated a hypothesis suggesting that many events that occur during the intrauterine life and early in infancy can influence the occurrence of many diseases that will develop in adulthood. This theory proposes that under-nutrition and other insult or adverse stimulus *in utero* and during infancy can permanently change the body’s structure, physiology and metabolism. The lasting or lifelong effects of under-nutrition will depend on the period in the development at which it occurs. The clues that led Barker to his conclusions started to be discovered when he was studying the temporal trends in the incidence of ischemic heart disease in England and Wales. Examining data found in The Hertfordshire records, collected in the beginning of the last century, he found that the rates of mortality by ischemic heart disease was much higher in children born in less affluent counties and mostly in those with low birth weight. After his initial findings a myriad of diseases have been found to be linked to low birth weight and under-nutrition *in utero* and in the neonatal period. These diseases were then nominated adult diseases with fetal origin. Epidemiological studies that led to these findings suggest that *in utero* and early postnatal life have critical importance for long-term programming of health and disease, opening unique chances for primary prevention of chronic diseases.

## Introduction

In order to understand what we weight from our intrauterine life until adulthood, we must understand our genes. It is supposed that at least 24.000 genes constitute the human blueprint and that over 250 of these genes may help determine our weight [1].

About 40.000 years ago, somewhere in the world, a Paleolithic couple emerged to become the great, great, great… grandparents of us all. Their genes still inhabit our cells, and we continue to pass them from one generation to the next, and these genes still shape our metabolic pathways. We must look to our Paleolithic ancestors to understand the modern-day problems of obesity, diabetes and many other diseases. We must look to these genes to know why the environment we have created is so aggressive to our health. We must understand how and why the genes that were advantageous in the past are so deleterious now [1].

Our ancestors were nomads. They used to travel long distances in search of food. The food sources were unreliable and no one ever knew exactly where or when they would get the next meal. When food was present, especially like fat and protein of animal origin, to store calories within the body was a very wise strategy [1].

Paleolithic men were possibly lean, muscular and strong. Their bodies evolved to withstand the danger that was everywhere. They used to have vigorous physical activity and insufficient food was a constant risk [1].

Women like the men used to be physically active and in order to supplement what men brought back home, they gathered nuts, berries, fruits, vegetables and roots. Obesity supposedly did not exist, because the food supply was so uncertain [1].

We cannot be certain, but possibly the Paleolithic diet was approximately 30 percent protein that came from fish and meat. We can certainly assume that the mammals our ancestors ate were also lean; they probably did not live in feedlots or graze on carefully managed pastures. They had to exert themselves to obtain food and to avoid becoming the meal of some other animal. So like the hunters who hunted them, their body composition was largely composed by muscles [1].

Our ancestors’ diet possibly consisted of up to 100 grams of fiber per day, what is 5–10 times higher than is typical today. Fat corresponded to approximately 20 percent and was mostly unsaturated since it used to come from nuts and seeds. Since the meat was also lean, Paleolithic diet was minimally composed by saturated fat [1].

Paleolithic men and women did not live long, possibly less than 20 years. If they survived birth and infancy, most died in what we consider today young adulthood. They were vulnerable to famine, predators, accidents and infections; the women faced all this plus the risk of childbirth. We can certainly assume that our ancestors did not have health problems obesity-related that plague us today. Because of their low fat intake, their blood vessels were probably free of fat deposits and stroke; heart attacks and high blood pressure were possibly rare. Diabetes and obesity were not known those days. Also, by not living so long, they would not have time to develop chronic diseases [1].

### Thrifty genes

The genes of our Paleolithic ancestors evolved for people who spent their days in constant physical activity and whose diet was low in calories and in saturated fat. Although, evolution selected genes that could support times of a poor food supply of a poor food supply, long winters and long times of recurrent droughts. These genes were called thrifty genes because they helped to maximize the amount of energy that could be obtained and stored from every consumed calorie [1,2].

One possible mechanism for accomplishing this was insulin resistance (IR) that was an adaptive condition for babies, before and after birth, in order to use few calories more efficiently. In times when food was more abundant, these genes would enable these babies to eat more and stock body fat for the future hard times that would certainly come. When food was scarce these genes would preserve those fat stores, slowing down metabolism and keeping the body’s energy reserves [1,2].

Thrifty genes were advantageous for life in the Paleolithic era. About 10.000 years ago, the world began to change. Many humans developed agriculture, domesticated animals, left behind their nomadic way of life, settled down and developed cities and civilizations. Famines became less frequent and the nutritional environment became altered. Humans started to eat more grains and consequently less fish, fruits and vegetables. Animals started to be raised in enclosed spaces and also became fatter. The saturated fat they contained was less favorable to the human metabolism and cardiovascular system [1,2].

It seems that these thrifty genes became less important in societies with better climate and abundant supplies. This helps to explain why obesity and diabetes for example, are more common in some parts of the world than in others [1,2].

### The scars of early life

In the 1980’s, Barker developed a hypothesis according which many nutritional events that occur during the intrauterine life and early in infancy will influence the development of adult diseases. This became the so called Barker hypothesis [3].

Lucas, proposed the term “programming” to describe the process by which an adverse event happening at a critical period of development, has long lasting or lifelong significance [4]. Fetal programming opened the field for extensive research into the fetal origin of adult diseases. The association between low birth weight (LBW), which reflects intrauterine nutritional status, and the development of adult diseases has been confirmed in many studies for type 2 diabetes (T2D), hypertension (HT) and ischemic heart diseases (IHD) [1-4]. These findings will be presented in this review.

Barker’s hypothesis suggests that under-nutrition and other insult or adverse stimulus *in utero* and during infancy can permanently change the body’s structure, physiology and metabolism. The lasting or lifelong effects of under-nutrition will depend on the period in the development at which it occurs. In early gestation it will reduce body’s size permanently, whereas in late gestation it will have deep effects on body form without necessarily reducing body size. Fetuses and neonates that are rapidly growing are more vulnerable to under-nutrition. These effects include altered gene expression, reduced cell numbers, imbalance between cell types, altered organ structure, pattern of hormonal release and hormonal responses [5]. Thus, the tendencies of our body to become obese, to develop T2D and many other diseases in the adulthood are affected by our genes, our early development and our lifestyle [1].

The clues that led Barker, a distinguished epidemiologist to formulate his hypothesis started to be discovered when he was studying the temporal trends in the incidence of IHD in England and Wales [5,6].

The incidence of IHD increased rapidly in the western world in the beginning of the 20^th^ century, and in the present days it has been growing in the so called developing countries such as China, India, Russia and in many eastern European countries. Such abrupt changes, in a so short time frame, could not be explained by genetic changes, and then the attention of the scientists was directed to the existing lifestyle in the industrialized countries. The relationship of IHD with obesity, smoking habit, high cholesterol levels and stress among many other factors have been well established [5,6].

In 1977, Forsdahl has found considerable variations in the rates of mortality from IHD in twenty Norwegian counties. He has suggested that these variations could not be explained by the current differences in standard of living existing then. Such differences did exist in the past as was shown by large variations in infant mortality. A significant positive correlation has been found between the county age-adjusted mortality from IHD in people aged between 40 and 69 years and county’s infant mortality relating to the early years in the same cohorts. His findings suggested that great poverty in childhood and adolescence followed by prosperity, was a risk factor for IHD [7].

Studying the geographic distribution of mortality by IHD, Barker has found that although the rise in IHD in England and Wales has been associated with increasing prosperity, paradoxically, mortality rates by IHD were higher in the least affluent areas. A strong geographical relation between IHD mortality rates in 1968–78 and infant mortality in 1921–25 was observed. IHD was found to be strongly correlated with both neonatal and postneonatal mortality rates. These findings led him also to suggest that poor nutrition in early life increases susceptibility to the effects of an affluent diet [3].

Barker concluded then that under-nutrition in women in childbearing age could be the origin of high rates of IHD in the next generation, since it would impair a woman’s ability to nourish her baby *in utero* and in early infancy [5,6].

### The Hertfordshire records

In order to test the hypothesis that IHD is programmed in utero, it was necessary to study people now, in middle and late life whose early growth had been recorded somewhere. Barker then undertook a search for medical records of babies born in the early 1900s, with the staff from the Medical Research Council of Britain. They searched archives and hospital record departments throughout the country. Many were found; some were in large collections preserved for many years, some had no more then a few hundred records that were kept by a clinic or a midwife. Some were found in lofts, sheds, garages, boiler rooms or flooded basements. Finally, in Hertfordshire, a county localized in the East region of England, just north of London, the appointments made by Ethel Margaret Burnside, the first county’s chief health visitor and lady inspector of midwives were found. She set up an army of trained nurses to attend women in childbearing age and to advise mothers about their babies health [5].

From 1911 onwards, when a woman in Hertfordshire had a baby, she was attended by a midwife that visited her home at regular intervals to get information about the baby’s health and development. The weight was recorded at birth and at one year of age, when visits ceased. From 1923 onwards the health visitors continued their visits until the child was five years old. The ledgers containing these information were maintained until 1945. They were found by the Medical Research Council in 1986 [5].

With the data found in Hertfordshire ledgers, Barker used records from England’s National Health Service to trace about 16.000 men and women who had been born in this county between 1911 and 1930. He then matched information about their current health status to the infant data that were collected by Burnside’s nurses. In 1989 when his study was published, 3.865 people had already died with ages ranging from 20 to 74 years. He observed that the mortality by IHD is almost two times more prevalent in those that had a birthweight ≤ 2.500 g when compared to those who had a birthweight ≥ 4.000 g. Barker discovered that men who had been small at birth, and who were still small at age one, were at the highest risk of presenting IHD. The mortality rates by any other disease had no relation to the birthweight [6].

Subsequent research throughout the world, has found similarly strong associations between LBW and IHD [8-10].

### Thrifty phenotype hypothesis or the small-baby-syndrome

The ‘thrifty phenotype’ hypothesis was proposed based on studies which showed that individuals who had a LBW (small babies) have an increased risk of developing symptoms of the metabolic syndrome (MS), T2D and cardiovascular diseases (CVD) later on [11]. This hypothesis, had the following two premises: 1) LBW is an indicator of maternal and, consequently, fetal under-nutrition, and 2) phenotypic characteristics that lead to a ‘saving’ of energy are beneficial for the individual in conditions of poor postnatal nutrition. Essentially, this hypothesis proposes that prenatal under-nutrition leads to decreased insulin secretion and, simultaneously, IR in the fetus which, in turn slows down prenatal weight gain. This phenotype results from active fetal adaptations and is preserved for the life span of affected individuals [11]. Accordingly, in later life such a phenotype must be ‘thrifty’ and help affected individuals to cope better with conditions of food shortage. However, under affluent conditions in modern western societies this advantage turns into a disadvantage and leads to the MS, T2D and CVD [11].

A small for gestational age (SGA) is a full term baby who is under 2.500 g at birth or born with a birth weight and/or length under two standard deviations (2 SDs) for the gestational age and sex of the population [12]. The determination of gestational age is generally difficult, being the most precise those performed with ultra-sound, while those assessed from the time of last normal menstrual period are deceivable [13,14].

The SGA babies can have their birth weight (SGA-w) affected, their birth length (SGA-l) or both (SGA-w/l). These subgroups achieve final height in different ways. SGA-w born children are mostly likely to achieve catch-up growth after the second year of life, while SGA-w/l children more frequently remain short in adulthood [15].

A growth retardation is a failure that can occur during the intrauterine development and is called intrauterine growth retardation (IUGR). If this condition is detected, both mother and fetus should undergo adequate monitoring by fetal biometry and doppler ultrasonography of uterine and fetal blood vessels [12].

The general incidence of SGA newborns is 3-10% [16-18]. In a study conducted in the USA in 2004 with 95.000 healthy newborns, 2.3% were SGA. The rate of LBW for the entire studied population (4.112.052) was 8.1% [19].

### Etiology of the small-baby-syndrome or small for gestational age

Most patients born SGA do not have a clear etiology for this condition to happen. Nevertheless, several maternal and fetal conditions have been identified as causative factors for the birth of a SGA baby.

Maternal factors can be related to insufficient substrate supply to the fetus during development due to many different causes such as reduced maternal food intake, maternal systemic diseases such as HT and diabetes, periodontal disease, abnormal placental function that can lead to an impaired utero-placental blood supply or disruption of the placental transfer, abruption, infarction or mal-development of the placenta. The majority of these factors can influence growth during the last trimester of pregnancy and result predominantly in IUGR that refers to poor growth of a baby while in the mother’s womb during pregnancy [20-23]. Other maternal contributing factors to SGA are: parity, ethnicity, delivery at age less than 16 and more than 35 years and previous history of SGA born children. Parents size seems to be less important on the baby’s birth weight [24].

The exposure of the fetus to a toxic intrauterine milieu caused by tobacco, alcohol consumption or illicit drugs abuse increase the risk of SGA or IUGR births. Smoking during pregnancy has the most significant influence with a relative risk of 3.24 [21,25].

Several fetal factors are related to the birth of a SGA baby, like some chromosomal anomalies such as gonadal disgenesy, Edward Syndrome, Turner Syndrome, Down Syndrome and Prader-Willi Syndrome [24].

The thrifty phenotype seems to be strongly associated with the birth of a SGA baby. Several mechanisms have been proposed to explain growth retardation of the fetus and the infant. The growth is assumed to be altered both quantitatively and qualitatively by a poor nutritional environment. Metabolic disturbances depend on the period of gestation in which a famine affected the mother and the children, as a Dutch SGA study showed in examining the population who suffered from famine during the Second World War [26,27]. If fetal exposure occurs during early pregnancy it will affect lipid metabolism, but if it occurs in late pregnancy, it will affect the glucose metabolism [26]. It is supposed that an inadequate development of pancreatic beta cell mass and their function are the link between poor fetal nutrition, IR and T2D later in life. A thrifty phenotype is adapted to survive in poor nutritional circumstances. Later in adulthood, abundant food intake and decreased energy expenditure lead towards obesity, glucose intolerance and HT among many other diseases, caused by epigenetic alterations that occurred during the intrauterine life [11,28,29].

How can it matter fifty or more years late that a person was born small? Nowadays, there is compelling evidence linking epigenetic factors to many human diseases. Epigenetic factors, by different types of reactions, could mediate the interplay between genes and environment resulting in activation or repression of genetic transcription, or even silencing the genetic transcription. The most important epigenetic reactions affecting genetic transcription are acetylation and methylation. These reactions occur mainly in the tail of histones that are proteins where DNA is wrapped. Brownlee et al. have demonstrated in human aortic endothelial cells, that excessive concentration of reactive oxygen species (ROS) can induce monomethylation of lysine from histone 3 increasing the expression of the subunit p65 of nuclear factor kappa beta. This reaction is responsible for the increased transcription of vascular cell adhesion molecule 1 and monocyte chemoattractant molecule 1 that are both related to diabetes, hypertension and other components of the MS [30,31].

Plagemann et al., have recently demonstrated in animal models that the neonatally acquired adipogenic and diabetogenic phenotype can probably be caused, at least in part, by over-nutrition in pre-and/or neonatal period, that can lead to alterations of DNA methylation patterns within the promoter regions of genes whose products are involved in the hypothalamic regulation of appetite, body weight and metabolism. In the promoter region of proopiomelanocortin (POMC), the most important anorexigenic neurohormone, neonatally overfed rats develop hypermethylation of activating transcription factor binding sites, in parallel with hypomethylation at an inhibitory transcription factor binding site. The promoter region of the hypothalamic insulin receptor gene promoter was found to be hypermethylated. These studies suggest that perinatal programming of long-term increased obesity and diabetes risk due to neonatal over-nutrition may occur via altered methylation patterns of the promoter regions of central nervous body weight-regulating neuropeptides and receptors [32-34].

### Consequences of the small-baby-syndrome or small for gestational age for newborns, infants and adolescents

During the newborn period SGA babies present increased risk of hypoglycemia, hypothermia, hypercoagulability, hyperbilirubinemia, hypotension, necrotizing enterocolitis, respiratory distress syndrome, lower Apgar scores, umbilical artery acidosis, more intubations and complications during delivery and approximately 20 times increased risk of neonatal death than babies born with an appropriate for gestational age (AGA) weight [24,35-37].

In the first two years of life, about 90–95% of children born SGA present catch-up growth [38]. More than 80% of SGA infants achieve catch-up growth during the first six months of life [39]. Ponderal index at birth is not related to postnatal catch-up growth in infants born SGA, but birth length and target (parental) height are important. The genetic influence on catch-up growth appears to start from the onset of childhood. For SGA children, being born short or becoming short during the first two years of life is similar in terms of risk for adult short stature [40].

In the childhood years, about 10% of children born SGA do not achieve catch-up growth after the second year of life and remain short (≤ 2 SDs) during childhood, adolescence and adulthood [38,41]. The risk of short final adult height was found to be five times higher for children with LBW and seven times higher for those with low birth length compared with children with normal birth size. At age 20, men and women were 4.50 cm and 3.94 cm, respectively, shorter than those born with AGA, and also have raised insulin and proinsulin levels which could be markers of early changes in insulin sensitivity [41].

Children born SGA seem to have modest independent effects on learning, cognition, and attention in adolescence [42]. They also have a greater risk of being psychosocially disadvantaged, less socially competent and present more behavioral difficulties due to impairments of neurocognitive and educational development and also specific adaptation difficulties towards short stature [43]. These children also present low scores of alertness, mood instability, significant differences in academic and professional achievements [44].

Children born SGA present early and rapid start of puberty; the amplitude of pubertal spurt is small, and they reach their final height earlier than children born with AGA. Girls have an advanced menarche by 5–10 months and boys have more genital alterations [38].

### Consequences of the small-baby-syndrome or small for gestational age for adults

After Barker’s findings of the strong associations between LBW and IHD it was suggested that many diseases of adulthood could have a fetal origin. Many subsequent studies have shown the association between LBW and a higher risk of developing several adult diseases.

In 1976, Ravelli et al., have conducted a historical cohort study of 300.000 19-year-old men exposed to the Dutch famine of 1944–45 and examined at military induction. They have found that outcomes were opposite depending on the time of exposure. During the last trimester of pregnancy and the first months of life, exposure to famine produced significantly lower obesity rates, suggesting that nutritional deprivation affected a critical period of development for adipose-tissue cellularity. During the first half of pregnancy, however, exposure resulted in significantly higher obesity rates consistent with the inference that nutritional deprivation affected the differentiation of hypothalamic centers regulating food intake and growth [45].

Many other conditions have been identified such as an increased risk of T2D [11,46,47] and IR with a decreased insulin-stimulated glucose uptake [48]; high death rates from IHD [49,50]; higher risk of developing MS [51-53]; CVD and HT independently of genetic factors, shared familial environment, and risk factors for HT in adulthood, including body mass index [54-57]; dyslipidemia with an atherogenic lipid profile [58-60] and obesity [61,62]. All these findings have been confirmed in many distinct populations such as in USA [63], Sweden [64], France [65], Norway [66] and Finland [67]. The association between LBW and T2D was found to be strong even after correction for many risk factors and it is independent of the degree of obesity and frequency and intensity of physical activity [68].

Epidemiological evidence of this casual relationship has been extended to many other diseases such as higher risk of breast cancer [69,70], end-stage renal disease mainly during the first 14 years of life [71,72], osteoporosis [73,74], spontaneous hypothyroidism [75], adult asthma [76], cardiac hypertrophy [77], depression [78], male reproductive health problems, including hypospadias, cryptorchidism and testicular cancer [38,79], liver cirrhosis [80], adult schizophrenia [81], adult hearing loss [82], polycystic ovary syndrome and precocious pubarche [83].

The phenotype that seems to be more strongly associated to higher risks of adult diseases is LBW followed by a fast catch-up growth [84-86].

## Conclusions

A clear phenomenological association has been demonstrated by many epidemiological studies between LBW and increased risk later in life, for many diseases such as IR, mortality by IHD, MS, T2D, CVD, HT, dyslipidemia, obesity, breast and testicular cancer, end-stage renal disease, osteoporosis, spontaneous hypothyroidism, adult asthma and hearing loss, cardiac hypertrophy, depression, liver cirrhosis, schizophrenia, polycystic ovary syndrome, precocious pubarche, hypospadias, cryptorchidism, low scores of alertness, mood instability, significant differences in academic and professional achievement. Probably, perinatally acquired alterations of DNA methylation patterns of gene promoters of central nervous regulators of body weight and metabolism play a key role in mediating these relationships. In conclusion, under-nutrition during neonatal life plays a critical role, beyond prenatal development, in the long-term programming of health and disease. This opens a variety of opportunities and challenges to primarily prevent chronic diseases such as stature deficits, endocrine, metabolic and neurodevelopmental disturbances during childhood and several diseases as those above mentioned, during adulthood.

This should be appropriately considered in future health care policies as well as research programs. Pre and neonatal under-nutrition should be avoided to prevent long-term deleterious consequences. Further studies are suggested to evaluate epigenomic mechanisms such as alterations of DNA methylation, that potentially underlie the increased risks for all these diseases.

## Abbreviations

IR: Insulin resistance; LBW: Low birth weight; T2D: Type 2 diabetes; HT: Hypertension; IHD: Ischemic heart diseases; MS: Metabolic syndrome; CVD: Cardiovascular disease; SGA: Small for gestational age; SGA-w: Small for gestational age with low birth weight; SGA-l: Small for gestational age with short length; SGA-w/l: Small for gestational age with low birth weight and length; IUGR: Intrauterine growth retardation; ROS: Reactive oxygen species; POMC: Proopiomelanocortin; AGA: Appropriate for gestational age.

## Competing interests

Both authors declare that they have no competing interests.

## Authors’ contributions

CAN and MBG drafted, reviewed and edited the manuscript. Both authors read and approved the final manuscript.
